# Association between emotional intelligence and academic success among undergraduates: A cross-sectional study in KUST, Pakistan

**DOI:** 10.1371/journal.pone.0219468

**Published:** 2019-07-10

**Authors:** Qaiser Suleman, Ishtiaq Hussain, Makhdoom Ali Syed, Rashida Parveen, Ishrat Siddiqa Lodhi, Ziarab Mahmood

**Affiliations:** 1 Department of Education & Psychology, Kohat University of Science & Technology, Kohat, Khyber Pakhtunkhwa, Pakistan; 2 Department of Education, University of Kotli, Kotli, Azad Jammu & Kashmir, Pakistan; 3 Department of Education, Fatima Jinnah Women University, Rawalpindi, Punjab, Pakistan; 4 Mohi-u-Din Islamic University Nerian Sharif, Azad Jammu & Kashmir, Pakistan; Universitat de Valencia, SPAIN

## Abstract

The study investigated the association between emotional intelligence and academic success among undergraduates of Kohat University of Science & Technology (KUST), Pakistan. A sample of 186 students who were enrolled during the semester Fall 2015 to Spring 2018 was selected through a random sampling technique. A cross-sectional, descriptive and correlational research methods were employed in this study. A standardized tool “Emotional Intelligence Scale” was employed for the collection of information from the undergraduates. Cumulative Grade Point Average (CGPA) of the students was considered as academic success. Data were collected through personal visits. Statistical tools i.e., simple percentage, mean, standard deviation, ANOVA, Pearson’s product-moment correlation and multiple linear regression were employed to reach the desired research outcomes. The findings revealed that there was a strong positive relationship (*r = 0*.*880*) between emotional intelligence and academic success among undergraduate students. The multiple linear regression analysis showed that self-development (*Beta = 0*.*296*), emotional stability (*Beta = 0*.*197*), managing relations (*Beta = 0*.*170*), altruistic behaviour (*Beta = 0*.*145*), and commitment (*Beta = 0*.*117*) predict academic success of undergraduates positively. The findings suggest that the emotional intelligence of the undergraduate students may be further improved so that their academic performance may further be enhanced.

## Introduction

Emotional intelligence is a conceptualization which progressively discussed in social psychology. Recently, emotional intelligence has been given much concentration in research especially in psychological research. The idea of emotional intelligence was introduced by Salovey and Mayer [1], who defined it as the capability of an individual to manage his own emotions and the emotions of other individuals, to differentiate among them and to utilize information to facilitate one’s activities, reasoning, and thinking. Afterward, the authors presented a revised and comprehensive definition of emotional intelligence as the capability to observe emotions, coordinate emotions to encourage thought, understand and control emotions to stimulate self-improvement [2]. Mayer, Caruso, and Salovey [1] are familiar with their incredible contribution to the rise of emotional intelligence. Subsequently, in 1995, the development of emotional intelligence construct commenced with the work of Daniel Goleman having an incredible contribution. Goleman [3] characterizes emotional intelligence as a collection of skills or capabilities i.e., having the ability to boost oneself and continue regardless of hindrances, to deal with compulsion and dissatisfaction, to manage one's mind-sets and keep sufferings from influencing the capability to think, to sympathize and to be optimistic. Goleman’s methodology is perceived as a mixed model of emotional intelligence which depicts a series of abilities and competencies comprising five key areas: self-awareness, social skills, self-regulation, motivation, and empathy [4]. Bar-On is another prominent psychologist in the field of emotional intelligence who has defined emotional intelligence as a variety of non-intellectual competencies, capabilities, and skills which have an impact on one’s capability to succeed in taking precedence over environmental pressures and demands [5].

Emotional intelligence may be characterized as the capability to identify, persist, control driving forces, communicate clearly, make incredible decisions, tackle issues, and perform with other individuals in such a way that makes companions and success [6]. These competencies enable a person to perceive and control emotions, ensure poise and dignity, formulate objectives, promote empathy, ensure conflict resolutions, and promote competencies essential for leadership and successful group participation [7]. Emotional intelligence is composed of significant parts of individual’s external as well as internal dealings, stress management abilities, mindset, personality, temperament adjustment and all these have significant influences on the academic accomplishment of university students [8]. Bradberry and Greaves [9] express that emotional intelligence is the individual’s capability, aptitude, recognition assignment, accurate assessment and controlling his senses against other individuals and groups. Emotional intelligence includes interpersonal intelligence and intrapersonal intelligence. Interpersonal intelligence is the external intelligence which an individual utilizes to comprehend and maintain relations with the other individuals. It is imperative for promoting characteristics like sympathy, empathy, and strengthening powerful relationships. On the other hand, intrapersonal intelligence is the internal intelligence which is used by an individual to know and understand himself which is necessary for self-awareness, self-inspiration, and self-regulation. The management of intrapersonal as well as interpersonal emotions is important for individuals’ academic and professional success. Individuals having higher emotional intelligence are more expected to regulate, understand, and control emotions excellently in themselves as well as in the other individuals [10].

Within the paradigm of emotional intelligence, three theories are considered the fundamentals of emotional intelligence [2–4, 11]. These theories have been presented in the last decade as an endeavor to explain the capabilities, attributes, and skills related to emotional intelligence. Model of emotional intelligence developed by Mayer and Salovey [2] is known as an ability model, concentrating on those constructs that stimulate intelligence through the understanding of emotions. In this model, emotional intelligence determines the potential for accomplishing proficiency of certain capabilities in the domain of emotional intelligence. Bar-On [11] presented a trait model of emotional intelligence which gauges emotional intelligence through five constructs such as intrapersonal skills, interpersonal skills, stress management, adaptability, and general mood. Interpersonal skills include the management of relationships with other individuals. Intrapersonal skills stress on individuals’ concentration and commitment and also the capability to make planning and complete independent ventures. Stress management abilities involve a person's capability to remain calm, use constructive managing strategies, and promote power supportive systems. Adaptability skills comprise of strong problem-solving aptitudes, flexibility and the capability to reframe issues and their resolutions. The general mood is a pointer of hopefulness, optimism, and resilience. Bar-On [5] expressed that emotionally intelligent individuals are commonly optimistic, adaptable, realistic, and effective in resolving issues and facing stressful situations without losing control. Goleman model of emotional intelligence [3–4] is a competency model which concentrates on the competencies of emotional intelligence that enable an individual to achieve accomplishment in the working place. Within the context of work performance, Goleman model is different from Bar-On [11] and Mayer and Salovey [2], who emphasize education and workplace products. Emotional intelligence with regard to work performance has been seemed to motivate others for solving problems, cooperating, and working to discover impartial approaches to ensure solutions for conflicts [12]. Goleman [4] additionally focused on emotional intelligence that comprises of five parts: identifying one’s emotions (self-awareness), managing them, inspiring self, recognizing emotions in others (empathy), and managing relationships.

Academic success or success is the product of instruction–the extent to which a student, educator, and institution have attained their educational aims. It is defined as the degree to which students attain the information, proficiencies, aptitudes, and skills that the teacher is going to teach or assign [13]. Academic success is viewed as one of the most significant conceptualizations within the domain of education that is intended to assess the accomplishment of the end goals of an individual’s success as well as the productivity of an educational system in future [14]. Emotional intelligence assumes a significant position within the realm of educational setting i.e., academic success, academic adaptation and psychological well-being of the students [15]. It is a significant determining factor of academic accomplishment in contemporary intensely stressful condition for students at each level of education [16]. The gap between endeavors for learning, powerful learning, and academic success can be covered by emotional intelligence [3]. Emotional intelligence has been considered having a direct association with the individual’s mental health [17] that ensures the individual’s wellbeing and happiness i.e., low-stress level, self-satisfaction [18].

Numerous investigations have revealed that there is a positive relationship between higher level of emotional intelligence and excellent academic success among adolescent students. The extensive body of research advocates that capabilities of emotional intelligence contribute to excellent performance [19–23]. In addition, emotional intelligence seems to have a substantial positive influence on institutional performance as well as academically weaker students [24–25]. Emotional intelligence’s abilities are considered four times more significant than IQ in deciding professional success and prestige. Emotional intelligence is a substantial predictor of performance in educational and other organizational settings [26]. Emotional skills, abilities, intelligence, and knowledge contribute to the enhancement of education, facilitation of students, instructors, faculty, and their professional development for the success of higher levels of accomplishment, career success, personal wellbeing, and leadership [27]. Hence, Goleman [3] recommended that emotional intelligence is a considerable predictor of academic success which is better than conventional measures of intelligence. Similarly, Bar-On [11] also perceives the impact of this non-intellectual capability in the success of a student’s life. He further recommends that the capability to manage one’s emotions, to enable to validate one’s emotions and to tackle issues of personal as well as interpersonal nature are essential for being educationally successful. Moreover, academic performance gives off an impression of being encouraged by having the capability to set personal goals and to be adequately hopeful and self-inspired to achieve them. Bar-On [28] indicates that emotionally intelligent individuals are committed, excited and eager in their life. Goleman [3] expresses that emotional intelligence represents 80% of all learning while cognitive capabilities represent about 20%. Although it is a strong claim, but yet it needs to be adequately investigated that to what degree emotional intelligence really correlates to academic performance.

Mayer, Salovey, and Caruso [29] proposed that emotional intelligence improves with the increasing of age. They also reported that as emotional intelligence expanded, academic success also improved and likewise, capabilities of communicating inspirational thoughts were also stimulated. Alternatively, as emotional intelligence diminished, oppositional behavior increased. Excellent emotional intelligence aptitudes were related to outstanding ability and capability to deal with one’s own feelings and the feelings of other individuals. Drago [30] assessed the association between academic success and emotional intelligence for nontraditional college students. A portion of the students was better equipped for the university environment on account of their intellectual capabilities. Hence, predictions of accomplishment and retention were possible due to the role played by emotional intelligence in academic success. Higher academic success was resulted due to the students’ abilities to understand, utilize, regulate and control their emotions effectively. Thus, fusing awareness of emotional intelligence into an academic program may contribute to the success of higher academic success by students and plausibly lead to the completion of their degree programs and retention. Zins, Elias, Greenberg, and Weissberg [31] affirmed that emotional and social learning might be the empowering factors that stimulate academic success. Research recommends that the "missing piece" in advancing academic accomplishment is instructive programming that blends social and emotional learning into the school’s curriculum [32]. Quality projects have been connected to enhanced academic performance through the advancement of students’ emotional intelligence capabilities [33]. Parker et al [34] concluded that the students who had achieved 80% or better were considered academically successful while students who had obtained 59% or less in their course work were regarded as academically unsuccessful. They noted that students who showed better academic performance also having higher emotional intelligence skills. They noted the difference between the groups and found that stress management was the main difference. Academically strong students exhibited increased focus which was an essential factor of stress management. Furthermore, they found that there were lesser differences in intrapersonal and adaptability ability.

## Conceptual framework

A conceptual framework is the understanding of researchers that how the study variables relate with each other. It presents a map for the investigation to be pursued. It describes systematically and logically the actions required to be taken during the research study through a picture or visual display [35]. In this cross-sectional study, a conceptual framework has been designed regarding the relationship between subdimensions of emotional intelligence and academic success in terms of Cumulative Grade Point Average (CGPA) (see Fig 1).

**Fig 1:** Conceptual framework of the Study. The Conceptual Framework shows the correlation model between subdimensions of emotional intelligence and academic success in terms of Cumulative Grade Point Average (CGPA) among undergraduate students.

## Methods and materials

### Population

This cross-sectional and correlative study was conducted in public sector university, Kohat University of Science & Technology (KUST) which is located in Kohat District of Khyber Pakhtunkhwa (Pakistan). It was established in 2001and was inaugurated by the former Governor of Khyber Pakhtunkhwa, Lt. Gen. Syed Iftikhar Hussain. It was awarded “W” the highest category by Higher Education Commission (HEC) of Pakistan. There are total seventeen different departments of social sciences, physical sciences, and biological sciences (see Table 1). The university aims to be one of the most responsive and energetic universities of the Khyber Pakhtunkhwa, providing outstanding educational opportunities for the graduates and undergraduates looking for the highest quality graduate, undergraduate, and unending professional or personal enhancement in all academic fields. The university offers quality and world-class education recognized by Higher Education Commission (HEC), Pakistan. The education at KUST offers a unique skill and experience to enable students to influence the society and workplace positively. It is one of the best universities in Pakistan to be acknowledged for its outstanding research activities. The University is trying to accomplish academic excellence through continuous enhancement of its teaching and research by providing students and faculty with a vibrant environment conducive for creation, dissemination, and assimilation of knowledge.

**Table 1:** Study population and sample size.

Faculties	Institutes/Departments	N	n (10% of N)
Social Sciences	Institute of Business Studies (IBS)	195	20
	Department of Education & Psychology (DEP)	02	00
	Department of English (DE)	262	26
	Department of Economics (DEc.)	72	07
	Department of Journalism & Mass Communication (DJMC)	17	02
	Department of Islamic & Pakistan Studies (DIPS)	00	00
	Department of Social Work & Sociology (DSWS)	55	06
Physical Sciences	Institute of Computing (IC)	334	33
	Department of Chemistry (DC)	173	17
	Department of Physics (DP)	95	10
	Institute of Numerical Sciences (INS)	82	08
Biological Sciences	Department of Microbiology (DM)	123	12
	Department of Biotech: & Genetic Engineering (DBDE)	121	12
	Department of Botany (DB)	07	01
	Department of Zoology (DZ)	121	12
	Department of Pharmacy (DPharm.)	197	20
**Total**	**17**	**1856**	**186**

All the undergraduate students of social sciences, physical sciences, and biological sciences enrolled during Fall 2015 to Spring 2018 constituted the population of the study. There are total seven departments in social sciences i.e., Institute of Business Studies, English, Education & Psychology, Journalism & Mass Communication, Economics, Islamic & Pakistan Studies, Social Work & Sociology. Similarly, there are total four departments in Physical Sciences i.e., Institute of Computing, Chemistry, Physics, and Institute of Numerical Sciences. In case of Biological Sciences, there are total five departments such as Microbiology, Biotechnology & Genetic Engineering, Botany, Zoology, and Pharmacy. In these departments, there were total 1856 undergraduates enrolled during the semester Fall 2015 to Spring 2018 (see Table 1).

### Sample and sampling technique

In this cross-sectional study, the sample was selected through simple random sampling technique from the aggregate of students enrolled in different semesters. From each department, 10% of the total undergraduate students were taken as a sample through Goldfish Bowl Method. According to the sampling outcomes, a total of 186 undergraduate students were selected from 1856 undergraduates (see Table 1).

### Research design and measurements

In the current study, a cross-sectional descriptive, quantitative and correlational research methods were used. Survey research design was used for gathering the required information from the undergraduates as it is more appropriate, authentic, economical and time-saving. Numerous researchers have described the advantages of survey research [36–39]. The surveys are widely used in research as reliable and authentic information can be gathered timeously at generally minimal effort and cost, particularly when contrasted with other research approaches i.e., ethnography [40].

In this cross-sectional study, data was collected from the participants through a standardized tool “Emotional Intelligence Scale” which is explained as under in detail:

#### Emotional Intelligence Scale (EIS)

Emotional Intelligence Scale (EIS) developed by Hyde, Pethe, and Dhar [41] was used for measuring the emotional intelligence of undergraduate students (see S1 Appendix). For this purpose, proper formal permission was sought from the authors of the EIS. Originally, Hyde, Pethe, and Dhar constructed a scale which was composed of 106 items but after statistical analysis, only 34 out of 106 items were found significant and that’s why the remaining items were excluded from the scale. To verify the reliability of the scale, they distributed the scale among a sample of 200 Indians executives and split half reliability was applied to their responses. The reliability coefficient and content validity were found 0.88 and 0.93 respectively. Besides, factor analysis was used on the scores and thus ten variables were found which establish the sub-measurements of the emotional intelligence scale. These ten sub-measurements along with items numbers are self-awareness (4 items), emotional stability (4 items), empathy (5 items), managing relations (4 items), integrity (3 items), self-motivation (6 items), commitment (2 items), self-development (2 items), value orientation (2 items), and altruistic behavior (2 items) (see Table 2). This scale has been constructed on five Point Likert Scale i.e., Strongly Agree, Agree, Undecided, Disagree, and Strongly Disagree and were scored as 5, 4, 3, 2, and 1 respectively. According to the Manual of Emotional Intelligence Scale, the total score obtained above 85 (mean score = 2.5) are regarded as “Above Average Emotionally Intelligent”. The total score obtained below 55 (mean score = 1.62) are considered as “Below Average Emotionally Intelligent” and the total scores achieved between 85–55 (mean score = 2.5–1.62) are rated as “Average Emotionally Intelligent”. In addition, the overall score of EIS was calculated by adding the mean scores of different subdimensions and then calculating their mean. Furthermore, the scale was translated into the Urdu language from English for a better understanding of the respondents. The various subdimensions of EIS are described as under:

**Table 2:** Subdimensions of Emotional Intelligence Scale (EIS).

S.#	Subdimensions of EIS	Item S. No.
1.	Self-Awareness	6, 12, 18, 29
2.	Emotional Stability	14, 19, 26, 28
3.	Empathy	9, 10, 15, 20, 25
4.	Managing Relations	1, 5, 11, 17
5.	Integrity	16, 27, 32
6.	Self-Motivation	2, 4, 7, 8, 31, 34
7.	Commitment	23, 24
8.	Self-Development	30, 33
9.	Value Orientation	21, 22
10.	Altruistic Behaviour	3, 13
**Total**		**34**

*Self-awareness* refers to the idea that a person acknowledges his own existence as an individual, different from other people, with private thoughts and considerations. *Empathy* is the capacity to perceive or comprehend the feelings and mentality of other individuals. *Self-motivation* is the capacity of an individual to stimulate and inspire his own personality, to examine a cause and the basic quality to achieve some goals. *Emotional stability* is the ability of the individual’s character to ensure the stability in even unpleasant and upsetting conditions. *Managing relations* is the inclination to move, support, motivate, influence, encourage and promote others while managing conflicts or utilizing consciousness of one's own emotions and that of others’ emotions to regulate relationships to accomplish productive and fruitful results. *Integrity* involves perceived consistency and regularity of activities, beliefs, convictions, methodologies, measures, and standards. Self-development refers to the individual obligations and liabilities for one’s own learning and advancement through a procedure of assessment, reflection, and execution. *Value Orientation* is the principle of good and bad that is accepted by a person or a society. *Commitment* refers to the responsibility or promise to something or someone and can be defined as individual obligation and responsibilities. *Altruistic behavior* refers to the behavior that is obliging and helpful for other people with little or no interest in being remunerated for one's efforts. An ethical principle which indicates that a moral duty of an individual to facilitate and help other individuals without considering his own benefits. a person having such a principle is known as Altruist [41].

#### Pilot testing

The Emotional Intelligence Scale has been validated through its developers on Indian executives, therefore, it was necessary to confirm its validity and reliability in Pakistani perspective. Secondly, it was translated into the Urdu language from English for a better understanding of the sample subjects. So, the instrument was pilot tested through 30 undergraduate students selected randomly from different departments of Kohat University of Science & Technology (KUST), Pakistan. Based on the findings of the pilot study, the instrument was found understandable and suitable in its Urdu version.

#### Validity of research instrument

Emotional Intelligence Scale was highly validated instrument widely used for measuring emotional intelligence of individuals, but it was necessary to confirm its validity with respect to Urdu version and research locality. So, the instrument was sent to four outstanding researchers of relevant fields for validation. Based on their review and feedback, it was found that the instrument in the Urdu version is highly validated in the research locality and only some minor changes were made in the language of the instrument.

#### Reliability of research instrument

In this cross-sectional study, test-retest reliability was used to confirm the reliability of the research instrument. It is calculated through a process where the same participants complete a survey at two different occasions to know to which degree the responses are stable. For this purpose, Pearson’s correlation is applied between the outcomes of pre-survey and post-survey. Generally, the correlation coefficient (r) values are regarded as good if r≥0.70 [42]. For this purpose, the instrument was distributed among 30 undergraduate students of different departments in Kohat University of Science & Technology, Pakistan and their responses were recorded. Similarly, after fifteen days, again the same instrument was distributed among the said undergraduate students and again their responses were measured. Then Pearson’s product-moment correlation was applied to the responses of the students recorded in pre-survey (test) and post-survey (retest). Table 3 presents the descriptive statistics and bivariate Pearson’s correlation between overall emotional intelligence as well as its subscales on pre-survey (test) and post-survey (retest). The analysis showed that there is a strong positive correlation (*r = 0*.*995*) between overall emotional intelligence on pre-survey and post-survey. Furthermore, there is strong positive correlation between all subdimensions of emotional intelligence on pre-survey and post-survey i.e., self-awareness (*r = 0*.*993*), empathy (*r = 0*.*972*), self-motivation (*r = 0*.*955*), emotional stability (*r = 0*.*959*), managing relations (*r = 0*.*989*), integrity (*r = 0*.*961*), self-development (*r = 0*.*995*), value orientation (*r = 0*.*992*), commitment (*r = 0*.*999*), and altruistic behaviour (*r = 0*.*995*). It undoubtedly indicates that the instrument has excellent reliability on the whole as well as with respect to all subdimensions.

**Table 3:** Pearson’s product-moment correlation analysis between the overall scores recorded in pre-survey and post-survey of emotional intelligent scale among undergraduate students.

Variables	n	Pre-Survey (Test)	Pre-Survey (Test-Retest)	Pearson’s Correlation	Sig
		Mean ± SD	Mean ± SD		
Overall Emotional Intelligence	30	30.51 ± 3.66	30.65 ± 3.45	0.995 *	< 0.01
Self-awareness	30	3.43 ± 0.656	3.44 ± 0.646	0.993 *	< 0.01
Empathy	30	2.33 ± 0.669	2.33 ± 0.669	0.972 *	< 0.01
Self-Motivation	30	3.24 ± 0.699	3.23 ± 0.652	0.955 *	< 0.01
Emotional Stability	30	2.54 ± 0.657	2.58 ± 0.627	0.959 *	< 0.01
Managing Relations	30	3.03 ± 0.739	3.07 ± 0.728	0.989 *	< 0.01
Integrity	30	3.17 ± 0.742	3.18 ± 0.704	0.961 *	< 0.01
Self-Development	30	3.28 ± 0.887	3.30 ± 0.867	0.995 *	< 0.01
Value Orientation	30	3.10 ± 0.995	3.13 ± 0.999	0.992 *	< 0.01
Commitment	30	2.99 ± 0.257	2.99 ± 0.255	0.999 *	< 0.01
Altruistic Behaviour	30	3.38 ± 0.888	3.40 ± 0.865	0.995*	< 0.01

*Correlation is significant at the 0.01 level (2-tailed)

**Reliability Strength:** 1.0 = Perfect Reliability; ≥0.9 = Excellent Reliability; ≥0.8<0.9 = Good Reliability; ≥0.7<0.8 = Acceptable Reliability; ≥0.6<0.7 = Questionable Reliability; ≥0.5<0.6 = Poor Reliability; <0.5 = Unacceptable Reliability; 0 = No Reliability

### Academic success (Cumulative Grade Point Average CGPA)

In the current study, academic success has been considered in terms of Cumulative Grade Point Average (CGPA). So, in order to record CGPA of the undergraduate students, a mandatory option was added in the demographic section of scale (see S1 Appendix). So, the demographic section was composed of different options i.e., name, the name of the department, gender, current semester, academic program, obtained CGPA, residence, parental education, parental income, and religion. In addition, the CGPA of the undergraduate students was also confirmed from the examination section of the university.

### Data collection

This cross-sectional study was officially approved by the Department of Education & Psychology, Kohat University of Science & Technology (KUST), Pakistan. The main purpose of this approval from the said department was to discuss and confirm the various aspects of the study including the feasibility as well as the applicability of the research study, the significance of the study, the ethical aspects and other related aspects. In addition, due to the involvement of human participants, ethical clearance for this cross-sectional study was also obtained from the same department. After the approval of the study from the aforementioned department, proper permission was sought from the heads of the departments of the said university in order to collect data from their undergraduate students. Then the data collection process was formally commenced on September 10, 2018 and completed on December 15, 2018. The researchers personally visited the respective sampled academic departments and met the Heads of the Departments for seeking formal permission for the collection of data. After getting permission, the researchers met the undergraduate students and they were explained the purpose of this investigation and its possible implications, facts, and consequences. After obtaining verbal informed consent from each undergraduate student, the research instrument was distributed among them for gathering the required information regarding emotional intelligence and CGPA. Due to extraordinary efforts by the researchers and follow up study, 100% response rate was achieved successfully from the actual sample subjects selected randomly.

### Data analysis

In order to analyze the data, descriptive statistics as well as inferential statistics were used. Descriptive statistics i.e., mean, standard deviation, skewness, and kurtosis were used for assessing the emotional intelligence and academic success of the undergraduates. A simple percentage was used for analyzing the demographic characteristics of the undergraduates. In case of inferential statistics, Pearson’s product-moment correlation was used to examine the association between emotional intelligence and academic success among undergraduates. Multiple linear regression and ANOVA were performed to find out the contribution of each subdimension of emotional intelligence in predicting academic success among undergraduate students.

## Results

### Participants’ demographic characteristics

In this cross-sectional study, 186 undergraduate students (male *n* = 119, female *n* = 67) participated on the request of researchers through formal permission. The statistical analysis presented in Table 4 depicts that 119(63.98%) of undergraduate students were males and 67(36.02%) were females. With respect to locality, 73(39.25%) undergraduates belonged to urban localities whereas 113(60.75%) heads belonged to rural localities. Regarding the age of undergraduate students, 33(17.74%) were in the age group 19 plus, 76(40.86%) were in age group 20 plus, 51(27.42%) were in age group 21 plus, and 26(13.98%) were in age group 22 plus. Among the undergraduates, 61(32.80%) were enrolled in social sciences, 68(36.56%) were enrolled in physical sciences, and 57(30.65%) were enrolled in biological sciences. With respect to academic semester, 28(15.05%) were enrolled in the 1^st^ semester, 24(12.90%) were enrolled in 2^nd^ semester, 56(30.11%) were enrolled in 3^rd^ semester, 41(22.04%) were enrolled in 4^th^ semester, and 37(19.89%) were enrolled in 5^th^ semester. In case of their residency, 119(63.98%) were day scholars and 67(36.02%) were boarder undergraduates. With respect to parental income level, 49(26.34%) undergraduates’ parental income level was Rs. 20000 ≤ Rs. 29000, 53(28.49%) undergraduates’ parental income level was Rs. 30000 ≤ Rs. 39000, 57(30.65%) undergraduates’ parents earned Rs. 40000 ≤ Rs. 49000, and 27(1452%) undergraduates’ parent has the income level equal to Rs. 50000 & Above. Regarding father educational level, it was found that 32(17.20%) undergraduates’ fathers were under matriculation, 27(14.52%) had matriculation, 26(13.98%) were intermediate passed, 53(28.49%) were Bachler degree holders, 46(24.73%) were Master degree holders, 2(01.08%) were MPhil degree holders, and no father was found having PhD degree. In case of mothers’ education level, 57(30.65%) undergraduates’ mothers were under matriculation, 22(11.83%) had matriculation, 26 (13.98%) were intermediate passed, 46(24.73%) were Bachler degree holders, 34(18.28%) were Master degree holders, 1(00.54%) were MPhil degree holders, and no mother was found having PhD degree. In case of the religion of the undergraduate students, 181(97.31%) had Islamic religion, 2(01.08%) were Hindus, 3(01.61%) were Christians, and 1(00.54%) belonged to other religions.

**Table 4:** Descriptive statistics of participants’ demographic characteristics (n = 186).

Characteristics	Categories	n (% age)
Gender	Male	119 (63.98%)
	Female	067 (36.02%)
Locality	Urban	073 (39.25%)
	Rural	113 (60.75%)
Age (in years)	19 +	033 (17.74%)
	20 +	076 (40.86%)
	21 +	051 (27.42%)
	22 +	026 (13.98%)
Enrolled in	Social Sciences	061 (32.80%)
	Physical Sciences	068 (36.56%)
	Biological Sciences	057 (30.65%)
Academic Semester	1^st^ Semester	028 (15.05%)
	2^nd^ Semester	024 (12.90%)
	3^rd^ Semester	056 (30.11%)
	4^th^ Semester	041 (22.04%)
	5^th^ Semester	037 (19.89%)
Residence	Day Scholar	119 (63.98%)
	Boarder	067 (36.02%)
Parental Income Level (per month)	Rs. 20000 ≤ Rs. 29000	049 (26.34%)
	Rs. 30000 ≤ Rs. 39000	053 (28.49%)
	Rs. 40000 ≤ Rs. 49000	057 (30.65%)
	Rs. 50000 & Above	027 (1452%)
Father’s Education	Under Matriculation	032 (17.20%)
	Matriculation	027 (14.52%)
	Intermediate	026 (13.98%)
	Bachler	053 (28.49%)
	Master	046 (24.73%)
	MPhil	002 (01.08%)
	PhD & Above	000 (00.00%)
Mother’s Education	Under Matriculation	057 (30.65%)
	Matriculation	022 (11.83%)
	Intermediate	026 (13.98%)
	Bachler	046 (24.73%)
	Master	034 (18.28%)
	MPhil	001 (00.54%)
	PhD & Above	000 (00.00%)
Religion	Islam	181 (97.31%)
	Hinduism	002 (01.08%)
	Christianity	003 (01.61%)
	Others	001 (00.54%)

### Descriptive statistics

Table 5 reflects the descriptive analysis of the emotional intelligence and academic success in the form of Cumulative Grade Point Average (CGPA) of undergraduate students enrolled in different disciplines of Social Sciences, Biological Sciences, and Physical Sciences during Semester Fall 2015 and Spring 2018. The results indicate that the academic success or success of undergraduate students was good as the mean CGPA was found 3.26 on the scale of 4.00 with a standard deviation of 0.783. The minimum and maximum CGPA were recorded as 1.80 and 4.00 respectively. To examine the emotional intelligence of undergraduate students, descriptive statistics regarding overall emotional intelligence revealed that they were found emotionally intelligent above average (*mean =* 3.43, SD = 0.510). The minimum and maximum mean scores of emotional intelligence of undergraduate students were found 2.09 and 4.48 respectively. The results show that undergraduate students were emotionally intelligent above average with all dimensions of emotional intelligence. The most rated subdimension of emotional intelligence was altruistic behaviour (*mean = 3*.*66*, *SD = 0*.*783)* followed by integrity (*mean = 3*.*57*, *SD = 0*.*723*) and self-awareness (*mean = 3*.*56*, *SD = 0*.*601)*. The other subscales of emotional intelligence were rated as managing relation *(mean = 3*.*51*, *SD = 0*.*640)*, value orientation *(mean = 3*.*50*, *SD = 0*.*786)*, self-development (Mean = 3.47, SD = 0.744), commitment *(mean = 3*.*38*, *SD = 0*.*428)*, and Self-motivation *(mean = 3*.*37*, *SD = 0*.*612)*, empathy *(mean = 3*.*32*, *SD = 0*.*532)*, and emotional stability (*mean = 2*.*91*, *SD = 0*.*640)*.

**Table 5:** Descriptive statistic of Cumulative Grade Point Average CGPA and emotional intelligence of undergraduate students.

Variables	N	Min	Max	Mean ± SD	SE	σ^2^	Skewness		Kurtosis	
							Statistic	SE	Statistic	SE
CGPA	186	1.80	4.00	3.26 **±** 0.783	0.027	0.134	−0.123	0.178	−0.603	0.355
OEI	186	2.09	4.48	3.43 ± 0.510	0.037	0.260	−0.116	0.178	−0.596	0.355
SA	186	2.00	5.00	3.56 ± 0.601	0.044	0.361	0.058	0.178	−0.166	0.355
E	186	1.80	4.80	3.32 ± 0.532	0.039	0.283	0.083	0.178	−0.160	0.355
SM	186	2.00	5.00	3.37 ± 0.612	0.045	0.374	0.151	0.178	−0.167	0.355
ES	186	1.00	5.50	2.91 ± 0.640	0.047	0.410	−0.272	0.178	1.055	0.355
MR	186	1.50	5.00	3.51 ± 0.640	0.047	0.410	−0.001	0.178	−0.247	0.355
I	186	1.67	5.00	3.57 ± 0.723	0.053	0.522	−0.109	0.178	−0.597	0.355
SD	186	1.50	5.00	3.47 ± 0.744	0.055	0.554	−0.197	0.178	−0.670	0.355
VO	186	1.50	5.00	3.50 ± 0.786	0.058	0.618	0.067	0.178	− 0.623	0.355
C	186	2.59	4.78	3.38 ± 0.428	0.031	0.183	0.026	0.178	−0.168	0.355
AB	186	2.00	5.00	3.66 ± 0.783	0.057	0.613	−0.077	0.178	−1.004	0.355

**Keys:** Min = Minimum; Max = Maximum; SD = Standard Deviation; SE = Standard Error; σ^2^ = variance; CGPA = Cumulative Grade Point Average; OEI = Overall Emotional Intelligence; SA = Self-awareness; E = Empathy; SM = Self-Motivation; ES = Emotional Stability; MR = Managing Relations; I = Integrity; SD = Self-Development; VO = Value Orientation; C = Commitment; AB = Altruistic Behaviour

### Inferential statistics

#### Pearson’s product-moment correlation analysis

**Null Hypothesis 1.** There is no significant relationship between emotional intelligence and academic success among undergraduates.

As presented in Table 6, a bivariate Pearson’s product-moment correlation was run to find out the relationship between emotional intelligence and academic success among undergraduate students. The value of correlations coefficient (*r*) was measured and found to be 0.880 which plainly indicates a strong significant (p<0.01) positive relationship between emotional intelligence and academic success. It shows that higher the emotional intelligence of undergraduate students than higher will be their academic success and so on. Therefore, the null hypothesis was rejected. The outcomes of the analysis have also been elaborated through scatterplot for better understanding (see Fig 2).

**Fig 2:** Correlation between emotional intelligence and academic success. The scatterplot clearly shows a significant positive relationship between emotional intelligence and academic success in terms of Cumulative Grade Points Average (CGPA) among undergraduate students of KUST.

**Table 6:** Bivariate pearson’s product-moment correlation (r) between the emotional intelligence and academic success among undergraduate students.

Variables	Emotional Intelligence	Academic Success (CGPA)
Emotional Intelligence	1.00	0.880 *
Academic Success (CGPA)	0.880 *	1.00

* Correlation is significant at 0.01 level (2-tailed).

**Correlation Strength:** r≥0.70 = Strong; 0.30≤ r ≤0.69 = Moderate; 0.01≤ r≤ 0.29 = Weak

**Null Hypothesis 2.** There is no significant relationship between the subdimensions of emotional intelligence and academic success among undergraduates.

Table 7 presents bivariate Pearson’s product-moment correlation between the subdimensions of emotional intelligence and academic success. The analysis showed that there is a strong positive correlation between three subdimensions of emotional intelligence and academic success i.e., managing relations (*r = 0*.*720)*, *integrity (r = 0*.*719*), and self-development (*r = 0*.*808*). Additionally, there is moderate positive correlation between seven subscales of emotional intelligence and academic success i.e., self-awareness (*r = 0*.*646*), empathy (*r = 0*.*617*), self-motivation (*r = 0*.*688*), emotional stability (*r = 0*.*696*), value orientation (*r = 0*.*663*), commitment (*r = 0*.*672*), and altruistic behaviour (*r = 0*.*656*). So, the null hypothesis was rejected. It means that emotionally intelligent undergraduate students will have excellent academic success. Additionally, the results have also been shown through scatterplots for more explanation (see Figs 3–5).

**Fig 3:** Correlation between the subdimensions of emotional intelligence and academic success. The scatterplots (a-d) clearly indicate the significant positive relationships among Self-awareness & CGPA; Empathy & CGPA; Self-Motivation & CGPA; and Emotional Stability & CGPA.

**Fig 4:** Correlation between the subdimensions of emotional intelligence and academic success. The scatterplots (a-d) plainly portray the significant positive relationship among Managing Relations & CGPA; Integrity & CGPA; Self-Development & CGPA; and Value Orientation & CGPA.

**Fig 5:** Correlation between the subdimensions of emotional intelligence and academic success. The scatterplots (a-b) undoubtedly represent the significant positive relationship among Commitment & CGPA; and Altruistic Behaviour & CGPA respectively.

**Table 7:** Pearson’s product-moment correlation between the subdimensions of emotional intelligence and academic success among undergraduate students.

Variables	SA	E	SM	ES	MR	I	SD	VO	C	AB	CGPA
**SA**	1.00										
**E**	0.518**	1.00									
**SM**	0.557**	0.570**	1.00								
**ES**	0.517**	0.591**	0.560**	1.00							
**MR**	0.545**	0.549**	0.564**	0.545**	1.00						
**I**	0.636**	0.588**	0.619**	0.531**	0.633**	1.00					
**SD**	0.674**	0.540**	0.666**	0.595**	0.638**	0.698**	1.00				
**VO**	0.592**	0.531**	0.620**	0.484**	0.581**	0.585**	0.661**	1.00			
**C**	0.612**	0.483**	0.560**	0.569**	0.529**	0.572**	0.634**	0.540**	1.00		
**AB**	0.559**	0.446**	0.583**	0.434**	0.524**	0.579**	0.605**	0.570**	0.464**	1.00	
**CGPA**	0.646**	0.617**	0.688**	0.696**	0.720**	0.719**	0.808**	0.663**	0.672**	0.656**	1.00

**Correlation is significant at 0.01 level (2-tailed).

* Correlation is significant at 0.05 level (2-tailed).

**Correlation Strength:** r≥0.70 = Strong; 0.30≤r≤0.69 = Moderate; 0.01 ≤r≤ 0.29 = Weak. **Key**: SA = Self-awareness; E = Empathy; SM = Self-Motivation; ES = Emotional Stability; MR = Managing Relations; I = Integrity; SD = Self-Development; VO = Value Orientation; C = Commitment; AB = Altruistic Behaviour; CGPA = Cumulative Grade Point Average

#### Multiple linear regression analysis

**Null Hypothesis 3.** Subdimensions of emotional intelligence have no significant effect in predicting academic success among undergraduates.

As depicted in Table 8, a multiple linear regression was done to find out the predictors of academic excellence among undergraduates. The value of ANOVA was computed and was found 70.178 which is statistically significant at 0.05. It means that the model is significant statistically. Additionally, the table indicates that the value of R square is 0.801 which depicts that 80% of the variance in academic excellence is substantially represented by the independent variables in the model. The multiple linear regression analysis revealed that among the subdimensions of emotional intelligence, five subdimensions were found substantial predictors and have a significant positive effect on academic success. Among these predictors, self-development (*Beta = 0*.*296*) was found the strongest predictor followed by emotional stability (*Beta = 0*.*197*), managing relations (*Beta = 0*.*170*), altruistic behaviour (*Beta = 0*.*145*), and commitment (*Beta = 0*.*117*) in defining academic success positively. On the contrary, self-awareness (*Beta = 0*.*041*), value orientation (*Beta = -0*.*031*), empathy (*Beta = 0*.*035*), self-motivation (*Beta = 0*.*047*), integrity (*Beta = 0*.*092*) and value orientation (*Beta = 0*.*043*) have no significant positive influence on academic success. Hence, the null hypothesis was rejected. It clearly indicates that self-development, emotional stability, managing relations, altruistic behavior, and commitment predict academic success positively among undergraduate students. With the increasing level of these subdimensions, academic success will be positively affected.

**Table 8:** Multiple linear regression to analyze the contribution of each independent variable (subdimensions of emotional intelligence) in predicting the dependent variable (Academic Success in terms of CGPA) among undergraduates (n = 186).

Academic Success in terms of Cumulative Grade Point Average (CGPA) (Dependent Variable)										
Model		Unstandardized Coefficients		Standardized Coefficients	*t*	*Sig*.	*R* Square	*F*	*Sig*.	*Durbin-Watson*
		*B*	*SE*	*β*						
Independent Variables	(Constant)	1.161	0.110		10.570	0.000	0.801	70.178	0.000	1.224
	SA	−0.019	0.031	−0.031	−0.593	0.554				
	E	0.024	0.033	0.035	0.732	0.465				
	SM	0.028	0.031	0.047	0.909	0.364				
	ES	0.112	0.027	0.197	4.105	0.000*				
	MR	0.098	0.028	0.170	3.458	0.001*				
	I	0.047	0.028	0.092	1.695	0.092				
	SD	0.145	0.029	0.296	4.926	0.000*				
	VO	0.020	0.023	0.043	0.842	0.401				
	C	0.100	0.042	0.117	2.378	0.019*				
	AB	0.068	0.022	0.145	3.088	0.002*				

* Significant Predictors

**Dependent Variable:** Cumulative Grade Point Average (CGPA). **Independent Variables:** SA = Self-awareness; E = Empathy; SM = Self-Motivation; ES = Emotional Stability; MR = Managing Relations; I = Integrity; SD = Self-Development; VO = Value Orientation; C = Commitment; AB = Altruistic Behaviour

## Discussion

The study examined the association between emotional intelligence and academic success in term of Cumulative Grade Point Average (CGPA) among undergraduates of Kohat University of Science & Technology Pakistan. For the successful conduction of this cross-sectional study, a correlative, descriptive and quantitative research methods were used. Mayer and Salovey [2] expressed that emotional intelligence is a conceptual framework that can influence emotional competencies and capabilities. There is an agreement among the majority of the scholars that there is a strong relationship between emotional intelligence and success in school, but this success requires a good IQ and the motivation of a person toward success [43]. Flattery [44] purported that learning involves coping with related emotions and learning contexts. Emotionally intelligent learners can cope with challenges emerged from the environment. Emotional intelligence acts as a background for understanding the association between cognition and emotions [29]. Globally, various research studies on the association between academic success and emotional intelligence have been conducted [21, 24, 45–53]. In the same way, the current study also examined the relationship between emotional intelligence and academic success among undergraduate students. Investigating emotional intelligence and academic performance of undergraduates, it is evident from the descriptive analysis that undergraduate students were emotionally intelligent on the whole. Based on the subdimensions of emotional intelligence, they were found emotionally intelligent above average with all subdimensions of emotional intelligence i.e., altruistic behavior, integrity, self-awareness, managing relation, emotional stability, value orientation, self-development, commitment, self-motivation, and empathy. In the case of academic performance, undergraduate students’ academic performance was found satisfactory.

In order to examine the association between emotional intelligence and academic success among undergraduate students, it is evident from the Pearson’s product-moment correlation analysis that there is a strong positive correlation between emotional intelligence and academic success among undergraduate students. It clearly indicates that if a student is emotionally intelligent, his academic performance will be excellent. In more simple words, emotional intelligence is directly related to academic success and higher the emotional intelligence, higher will be the academic success and vice versa. It can be assumed that for better academic performance, students’ emotional intelligence should be enhanced. According to Greenleaf [43], when the emotional state of a learner is positive, the organization of cognitive memory can be stimulated, and the learner will grow intellectually. Conversely, negative emotions hinder learners from connecting their learning to the task at hand and from creating meaning and relevance. In order to explore the contribution of each dimension of emotional intelligence in predicting academic success of undergraduate students, multiple linear regression was applied. The outcomes of regression analysis explored that among the subdimensions of emotional intelligence, five subdimensions were confirmed significant predictors and have a significant positive effect on the academic success of the students. Among these predictors, self-development was rated to be the strongest predictor followed by emotional stability, managing relations, altruistic behavior, and commitment in defining academic success positively. With the increasing level of these subdimensions, academic success will be positively affected. In contrast, self-awareness, empathy, self-motivation, value orientation, empathy, self-motivation, integrity and value orientation have no significant positive influence on academic success.

The findings of the study are consistent with the findings of Petrides, Frederickson, and Furnham [24] who confirmed that emotional intelligence has a substantial positive connection with academic performance as well as cognitive ability. In addition, they noted that emotional intelligence is moderately correlated with academic success and intellectual ability. Similarly, Schutte et al [51] affirmed that emotional intelligence is an outstanding predictor of academic excellence in terms of Grade Point Average among undergraduates. Correspondingly, Chew, Zain, and Hassan [54] found that emotional intelligence is significantly correlated with the academic performance of final year students. Students who were more emotionally intelligent showed better performance in both the continuous assessments and the final professional examination. The total emotional intelligence score was a significant predictor of good overall continues assessments (CA) and a negative predictor of the poor result in overall continues assessments. Shahinzadeh and Barkhordari [55] also concluded that there is a meaningful and direct relationship between students’ emotional intelligence and mathematics success. Parker, Summerfeldt, Hogan, and Majeski [21] concluded that the highly successful students achieved higher scores as compared to the unsuccessful group on three subcategories of emotional intelligence such as stress management, intrapersonal ability, and adaptability. The outcomes of the study are also supported by the findings of Fallahzadeh [8] who affirmed a considerable association between emotional intelligence and academic performance although findings showed a significant association between two subdimensions of emotional intelligence and academic performance. Ranjbar, Khademi, and Areshtanab [49] found a weak correlation between educational success and emotional intelligence. They noted that the association of these variables may be influenced by other variables in this setting, so it needs further investigation in this area.

Conversely, the findings of the study negate the findings of Zirak and Ahmadian [56] who concluded that there is no significant positive association between emotional intelligence and academic success. Likewise, Azimifar [57] also revealed contradictory results that there is no statistically significant correlation between students’ scores and the achievement tests. More surprisingly, Shah, Sanisara, Mehta, and Vaghela [52] found that there is a negative association between academic success and emotional intelligence. Accordingly, academic success is negatively affected by higher emotional intelligence. Similarly, Olatoye, Akintunde, and Yakasai [48] and Gilani, Waheed, Saleem and Shaukat [46] also found a negative insignificant association between emotional intelligence and academic success. Based on the aforementioned research outcomes, it can be assumed that there is no unique agreement among the researchers on the association between emotional intelligence and academic success. Therefore, there is a need for further investigation on the association between these two variables.

## Limitations

Every research study has certain shortcomings, limitations, or drawbacks which may affect the outcomes of the research study. This study has some shortcomings and limitations. Firstly, the problem has been investigated through only quantitative research methodology and therefore, the same problem may be investigated by applying a mixed method research methodology i.e., quantitative as well as qualitative methodology in future research. Secondly, the data was collected through a standardized tool and there is a possibility of a slight difference in the findings if the data may be collected through a self-developed measuring instrument. Thirdly, different demographic variables i.e., age, gender, academic semester, locality, parental education, parental income, nature of family, etc. are the important variables which may affect the outcomes of the study, but these variables were not considered in this study. Therefore, if someone wants to conduct such type of study with respect to these demographic variables, then it is possible that the outcomes may slightly differ from the findings of the current study. So, this shortcoming may be overcome through future research study with these demographic variables. Fourthly, only CGPA as a representation of academic success was considered in this study which is a limitation of the study. Therefore, other domains of academic success may be considered in the future research study. Fifthly, this cross-sectional study has been conducted in only one public sector university of Khyber Pakhtunkhwa. There is a possibility that the results may differ to some extent if the same study may be conducted in all universities of Khyber Pakhtunkhwa. Therefore, the gathering of information from all the universities of Khyber Pakhtunkhwa with bigger sample size will overcome this limitation. In this way, it will provide a broad, comprehensive and ample representation of the actual scenario.

## Conclusions

Conclusively, undergraduate students were found emotionally intelligent. They were found emotionally intelligent with respect to all subdimensions of emotional intelligence i.e., self-awareness, self-development, integrity, managing relation, self-motivation, emotional stability, value orientation, commitment, altruistic behavior, and empathy. Academically, their performance was found satisfactory. Regarding the relationship between emotional intelligence and academic success, a strong positive relationship was found between emotional intelligence and academic success in term of Cumulative Grade Point Average. In case of subdimensions, a significant positive relationship was found between all the subdimensions of emotional intelligence and academic success. It evidently shows that higher the level of emotional intelligence, higher will be the academic success. In addition, five subdimensions were found significant predictors of academic success and have a significant positive influence on the students’ academic success. Among these predictors, self-development was rated to be the strongest predictor of academic success followed by emotional stability, managing relations, altruistic behavior, and commitment. It undoubtedly reveals that with the increasing level of these subdimensions, academic success will be positively affected. In nutshell, there was a strong positive correlation between emotional intelligence and academic success. Also, emotional intelligence can predict students' academic success.

The findings suggest that emotional intelligence is closely linked with high academic success. Hence, it is necessary to accentuate those practices which promote emotional intelligence and commitment among undergraduate students. The curriculum designers and developers should integrate emotional intelligence into the curriculum at each level in order to produce emotionally intelligent students. The educators should teach emotional intelligence competencies at each level to enable students to understand themselves and other individuals, to manage their own emotions and emotions of others, to take care of others and know how to perform. In this way, the students’ academic performance will be enhanced. At each level, various programs, conferences, and seminars on emotional intelligence should be arranged to educators in order to provide the necessary information for enhancing the emotional intelligence of their students.

## Supporting information

S1 Appendix Emotional Intelligence Scale (EIS). (PDF)

S1 Data Set Data set regarding scores on the emotional intelligence scale of undergraduate students. (XLSX)

S2 Data Set Data Set regarding data for calculating test-retest reliability of emotional intelligence scale. (XLSX)
